This article has been retracted.

# Deep Transfer Learning-Based Breast Cancer Detection and Classification Model Using Photoacoustic Multimodal Images

**DOI:** 10.1155/2022/3714422

**Published:** 2022-05-05

**Authors:** Maha M. Althobaiti, Amal Adnan Ashour, Nada A. Alhindi, Asim Althobaiti, Romany F. Mansour, Deepak Gupta, Ashish Khanna

**Affiliations:** ^1^Department of Computer Science, College of Computing and Information Technology, Taif University, P.O.Box 11099, Taif 21944, Saudi Arabia; ^2^Department of Oral & Maxillofacial Surgery and Diagnostic Sciences, Faculty of Dentistry, Taif University, P.O. Box 11099, Taif 21944, Saudi Arabia; ^3^Oral Diagnostic Sciences Department, Faculty of Dentistry, King Abdulaziz University, Jeddah, Saudi Arabia; ^4^Regional Laboratory and Blood Bank, Taif Health, Taif, Saudi Arabia; ^5^Department of Mathematics, Faculty of Science, New Valley University, El-Kharga 72511, Egypt; ^6^Department of Computer Science & Engineering, Maharaja Agrasen Institute of Technology, Delhi, India

## Abstract

The rapid development of technologies in biomedical research has enriched and broadened the range of medical equipment. Magnetic resonance imaging, ultrasonic imaging, and optical imaging have been discovered by diverse research communities to design multimodal systems, which is essential for biomedical applications. One of the important tools is photoacoustic multimodal imaging (PAMI) which combines the concepts of optics and ultrasonic systems. At the same time, earlier detection of breast cancer becomes essential to reduce mortality. The recent advancements of deep learning (DL) models enable detection and classification the breast cancer using biomedical images. This article introduces a novel social engineering optimization with deep transfer learning-based breast cancer detection and classification (SEODTL-BDC) model using PAI. The intention of the SEODTL-BDC technique is to detect and categorize the presence of breast cancer using ultrasound images. Primarily, bilateral filtering (BF) is applied as an image preprocessing technique to remove noise. Besides, a lightweight LEDNet model is employed for the segmentation of biomedical images. In addition, residual network (ResNet-18) model can be utilized as a feature extractor. Finally, SEO with recurrent neural network (RNN) model, named SEO-RNN classifier, is applied to allot proper class labels to the biomedical images. The performance validation of the SEODTL-BDC technique is carried out using benchmark dataset and the experimental outcomes pointed out the supremacy of the SEODTL-BDC approach over the existing methods.

## 1. Introduction

Multimodal imaging plays a significant role in the healthcare of different diseases by enhancing the clinician's capability to implement surveillance, monitoring, diagnosis, staging, therapy guidance, planning, evaluating recurrence, and screening therapy efficacy [1]. The multimodal imaging system has been extensively employed in clinical practice and medical research [2], namely, tumor resection surgeries, cardiovascular disease, neuropsychiatric disease, and Alzheimer's. Photoacoustic imaging (PAI) is a hybrid biomedical imaging system that exploits optical and acoustical features [3]. PA imaging was assessed as a clinical and preclinical imaging technique in the biomedical fields. PA imaging depends on the PA effect. Once a pulsed laser using a pulse width of nanosecond illuminates a targeted object, a PA wave could be consequently induced object subsequent relaxation and thermoelastic expansion [4]. An ultrasound (US) transducer identifies the PA wave, and an image is recreated by using an imaging system. PAI is current example of the effective rise of optical imaging modality. PAI uses the absorption features of exogenous or endogenous biomarkers for generating targeted image contrast with a wide-ranging penetration depth and spatial resolution [5].  Figure 1 illustrates the process of PAI.

The rich absorption data that PAI offers will be complemented well by an imaging modality that provides scattering data in detail. Depending on the way image is formed, PAI is split into two major classes: photoacoustic microscopy (PAM) that employs focused-based image formation and photoacoustic tomography (PAT) that employs reconstruction-based image formation [6]. Usually, in PAT, a wide-ranging unfocused excitation beam is collectively utilized with an array of ultrasonic detector that measures the ultrasound wave in various locations [7]. It provides field of view (FOV) images and is utilized in applications like breast cancer studies and whole-body imaging of small animals. Mammography is utilized very much for earlier screening and detection of breast cancer over the last few years, but reading mammography is a labor-intensive task for radiotherapists, who cannot offer reliable outcomes between readings [8]. The readings are based on subjective, training, and experience criteria. Computer-aided diagnosis (CAD) system assists radiotherapist in interpreting sonography for mass classification and detection. The usage of machine learning (ML) was quickly increasing in the field of medical imaging, including radiomics, medical image analysis, and CAD. Lately, ML field named deep learning (DL) appeared in the computer vision fields and become more common in various areas [9]. It started from an event in late 2012, once a DL method depends on a convolution neural network (CNN) won an overwhelming victory in the better-known worldwide CV competition, ImageNet Classification. Thereafter, researchers in almost every field, including medicinal imaging, have actively started contributing to the increasing area of DL [10–13].

This article introduces a novel social engineering optimization with deep transfer learning-based breast cancer detection and classification (SEODTL-BDC) model using PAI. The SEODTL-BDC technique involves bilateral filtering (BF) as an image preprocessing technique to remove noise. Moreover, a lightweight LEDNet model is employed for the segmentation of biomedical images. Also, residual network (ResNet-18) model can be utilized as a feature extractor. Furthermore, SEO with recurrent neural network (RNN) model is applied for image classification. In order to demonstrate the enhanced outcomes of the SEODTL-BDC model, a series of simulations can be performed using benchmark dataset.

## 2. Literature Review

Manwar et al. [14] presented an approach-based DL method for virtually increasing the MPE to improve the signal-to-noise ratio of deep structure from the brain tissues. The presented approach estimated in vivo sheep brain imaging research. Then, approach could enable medical translation of photoacoustic method in brain imaging, particularly in transfontanelle brain imaging in neonates. Ma et al. [15] developed an approach for automatically generating breast mathematical models for PAI. The distinct kinds of tissue are automatically extracted initially by applying DL and other techniques from mammography. Later, the tissue is integrated with arithmetical set operation for generating a breast image afterward being allocated optical and acoustic parameters.

Zhang et al. [16] investigated the DL methods in emerging tomography for breast cancer diagnosis. Especially, we utilized a preprocessing method for enhancing the uniformity and quality of input breast cancer images and a transfer learning (TL) technique to accomplish good classification accuracy. Lan et al. [17] introduced a CNN architecture Y-Net: a CNN framework for reconstructing the first PA pressure distribution by improving raw data and beamformed images. The network integrase 2 encoders with one decoder path optimally use data from beamformed images and raw information. Jabeen et al. [18] introduced an architecture for breast cancer classification in ultrasound images which applies DL and fusion of the optimal chosen features. The presented method is classified into the following: (i) data augmentation is implemented for increasing the size of new data set for learning of CNN model; (ii) a pretrained DarkNet-53 architecture is taken into account, and the output layer is adapted on the basis of data set class.

Zhu et al. [19] developed an automated system for categorizing thyroid and breast cancers in ultrasound images with DCNN. Particularly, we proposed a generic DCNN framework using TL and the similar structural parameter settings for training model to thyroid and breast lesions (TNet and BNet) correspondingly and test the feasibility of generic model using ultrasound images gathered from medical practice. Ha et al. [20] examined the capability of CNN to forecast axillary lymph node metastasis with primary breast cancer ultrasound (US) images. The CNN has been executed completely of 3 × 3 convolution kernels and linear layer. Feature maps were downsampled with strided convolution.

## 3. The Proposed Model

In this study, a novel SEODTL-BDC technique has been developed for the detection and classification of breast cancer utilizing ultrasound images. The proposed SEODTL-BDC technique encompasses a series of subprocesses, namely, BF-based preprocessing, LEDNet-based segmentation, ResNet-18-based feature extraction, RNN-based classification, and SEO-based hyperparameter tuning. The detailed working of every module involved in the SEODTL-BDC technique is elaborated in the following.  Figure 2 depicts the overall process of SEODTL-BDC technique.

### 3.1. Preprocessing

In this study, BF technique is used as an image preprocessing tool. It smoothens the images without changing the edges, through a nonlinear integration of the closing value of an image. The presented approach is simple, local, and noniterative. It integrates gray levels, based on the photometric similarity and geometric proximity. It selects closer values to distance values in range and domain. In contradiction of filter functioning in 3 individual color bands, a 2-sided filter enforces the fundamental perception metrics in the CIE-Lab color space, smoothens the color, and preserves the edge to suit human perception [21].

### 3.2. Image Segmentation: LEDNet Model

LEDNet follows an encoding-decoding infrastructure. It utilizes an asymmetric sequential infrastructure, whereas encoding produces downsampled feature map, and following decoding adapts APN which upsamples the feature map for matching input resolution. Also SS-nbt unit, the encoding also contains downsampling unit that is carried out by stacking 2 parallel resultants of single 3 × 3 convolutional with stride 2 and max-pooling. The downsampling allows very deeper network for gathering contexts but is simultaneously used for reducing computation. In addition, the procedure of dilated convolution permits infrastructure to take huge receptive domain, resulting in an enhancement in accuracy. Related to utilize of superior kernel size, this approach was established to enhance efficiency with respect to computational cost and parameters.

Simulated by attention process [22], the decoding design APN for performing dense evaluation utilizes spatial-wise attention. For increasing receptive domain, the APN adapts a pyramid attention element that combines features in 3 distinct pyramid scales. It is initial employ 3 × 3, 5 × 5, and 7 × 7 convolutional with stride 2. Afterward, the pyramid infrastructure fuses data of distinct scales step-by-step that is integrate neighbor scales of context accurately. As higher-level feature map is smaller resolution, utilizing huge kernel size does not bring excess computation burden. Afterward, a 1 × 1 convolutional was executed to the resultant of encoding; next, the convolution feature map is pixel-wisely multiplied by pyramid attention feature. In order to improve efficiency, a global average pooling branch was established for integrating global context prior attention. Eventually, an upsampling unit was utilized for matching the resolution of input images.

### 3.3. Feature Extraction: ResNet-18 Model

During feature extraction process, the segmented image is passed as to ResNet-18 technique to identify the lesion regions in the ultrasound images [23]. For extracting deep features from input images, a deep CNN was needed that trained. But once the model is deep, the degradation issue is prone to take place. While the method obtains very deeper, the model performance will not enhance but reduce. The residual block (RB) that is stacked from the models is the core of ResNet. Different from traditional CNN stacked by convolution and pooling layers, all the RBs are comprised of 2 convolution layers and short connections. Now, *x* denotes the input signal, and *F* (*x*) represents the resultant of RB beforehand the 2^nd^ layer activation function. When W1 and W2 represent the weight of 1st and 2nd layer of RB, correspondingly, *F* (*x*) is determined by *F* (*x*) = W2f (W1X). In the RB, activation function *f* employs ReLU. Therefore, the last outcome of RB is *f* (*F* (*x*) + *x*).

Assume the target output of RB was equivalent to the input *x* that is easily viewed in a DL architecture. On the other hand, we needed to enhance *x* to *F* (*x*) = *x* from traditional CNN without shortcut connection. Here, it can be trained an 18-layer CNN (ResNet-18) comprised of eight RBs, 7 × 7 convolution layers, one fully connected layer, and two pooling layers for realizing the automated classification of TUSP images afterward resizing and padding. Also, all the RBs are comprised of two 3 × 3 convolution layers.

### 3.4. Image Classification: Optimal RNN Model

At the final stage, the SEO-RNN model can be applied for the detection and classification of breast cancer using ultrasound images. It is a preassumption in a conventional NN that each input and output are independent of one another. Nevertheless, this assumption is not true in several applications, especially those that utilize series data, like speech recognition tasks. Different from a conventional NN, RNN generates output dependent on the prior state calculated and repeatedly implements a similar task for sequential components. In another word, RNN benefitted from having a memory that stores formerly estimated data. RNN is commonly utilized for language modeling and showed greater potential in natural language processing tasks [24]. The possibility is given in the following:

(1) $$\begin{array}{c} P\left(w_{1},w_{m}\right)=\overset{m}{\underset{i=1}{\prod }}P\left(\left.w_{i}\right|w_{1},w_{i}-1\right). \end{array}$$

Consider *x*_*t*_ and *h*_*t*_ represent the input and hidden states at timestamp *t*, correspondingly. The output *y*_*t*_ at timestamp *t* is determined by

(2) $$\begin{array}{c} y_{t}=soft\max\left(Vh_{t}\right), \end{array}$$

whereas *V* denotes the weight matrix of output layer.

*h*_*t*_ represents the memory of network and is estimated according to the preceding hidden layer and the input at the existing step: *h*_*t*_ = *f*(*Ux*_*t*_ + *Wh*_*t*−1_) . *U* and *W* represent weight matrix for the input and hidden states, correspondingly. Usually, the activation function *f* is a nonlinearity, namely, tanh, ReLU, or sigmoid. In RNN, the overall amount of variables is reduced in comparison to FFNN as each parameter is shared between each step. Hence, for distinct inputs, a similar task is implemented at every step.

For optimally tuning, the hyperparameters involved in the RNN model, the SEO algorithm can be utilized. SEO algorithm is a two-solution based metaheuristic proposed by Fard et al. [25]. The subsequent step describes the algorithm. The metaheuristic is initialized by fitness values and two random solutions, and the optimal solution takes the role of defender and attacker. Here, a solution is called a person, and the variable of solution is called traits. In *N*_var_-dimension optimization problem, a person is initialized arbitrarily as array of size 1×*N*_var_, represented by

(3) $$\begin{array}{c} \text{person}=\left[X_{1},X_{2},\cdots ,X_{N_{\mathrm{var}}}\right]. \end{array}$$

Afterward, the solution was initialized, and their fitness value has estimated. The steps mimic the retraining and training of the attackers from the defenders. Now, the attackers attempt to test on all the variables (trait) of defender to recognize the effective trait. Next, *α* percentage of attacker trait is chosen arbitrarily and replaced with the similar trait of the defender as

(4) $$\begin{array}{c} N_{\text{Train}}=\text{round}\left\{\alpha \times N_{\mathrm{var}}\right\}, \end{array}$$

whereas *α* indicates the percentage of chosen traits, and *N*_var_ indicates the overall amount of traits in a person. *N*_rain_ shows the count of attacker traits that exchanged with similar arbitrary traits of defenders. Firstly, the attacker directly abuses the defender to attain the purpose as follows.

(5) $$\begin{array}{c} \text{de}{\text{f}}_{\text{new}}=\text{de}{\text{f}}_{\text{old}}\times \left(1-sin\beta \times r_{1}\right)+\frac{\left(\text{de}{\text{f}}_{\text{old}}+\text{att}\right)}{2}\times \sin\beta \times r_{2}, \end{array}$$

whereas def_new_ and def_old_ denote the new and present locations of the defender, correspondingly. att signifies the existing location of attackers. *β* indicates the rate of spotting an attack. *r*_1_ and *r*_2_ are the initialized arbitrarily within [0, 1].

At the time of phishing, the attacker pretended to attack the defender thus the defender changed to a novel location whereby the attacker needs it to be.

(6) $$\begin{array}{c} \text{de}{\text{f}}_{\text{new}}^{1}=\text{att}\times \left(1-\sin\beta \times r_{1}\right)+\frac{\left(\text{de}{\text{f}}_{\text{old}}+\text{att}\right)}{2}\times \sin\beta \times r_{2}, \end{array}$$

(7) $$\begin{array}{c} \text{de}{\text{f}}_{\text{new}}^{2}=\text{de}{\text{f}}_{0}\left|d\right.\times \left(1-\sin\left(\frac{\pi }{2}-\beta \right)\times r_{1}\right)+\frac{\left(\text{de}{\text{f}}_{\text{old}}\right.+\left(\text{att}\right)}{2}\times \sin\left(\frac{\pi }{2}-\beta \right)\times r_{2}. \end{array}$$

During diversion theft process, the attacker guides the defender to a novel location from deception as follows:

(8) $$\begin{array}{c} def_{new}=def_{\text{old}}\times \left(1-\sin\beta \times r_{1}\right)+\frac{\left(def_{\text{old}}\right.+\left(\text{att}\times r_{2}\right)\times \sin\left(\pi /2-\beta \right)}{2}\times \sin\beta \times r_{3}. \end{array}$$

In pretext, the attacker traps the defender to defeat it. One novel solution is generated as follows:

(9) $$\begin{array}{c} \text{de}{\text{f}}_{\text{new}}=\left(\text{de}{\text{f}}_{\text{old}}\times r_{1}\times \sin\left(\frac{\pi }{2}-\beta \right)\right)\times \left(1-\sin\beta \times r_{2}\right)+\frac{\left(\text{de}{\text{f}}_{\text{old}}\times r_{3}\times \sin\left(\pi /2-\beta \right)\right)+\text{att}}{2}\times \sin\beta \times r_{4}. \end{array}$$

In which *r*_1_, *r*_2_, *r*_3_, and *r*_4_ are arbitrary values within [0, 1].

While responding to attacks, a novel location of the defender is estimated and compared to its older location. Furthermore, the optimum location for the defender is selected. When the novel location of the defender has superior to the attacker, the attacker becomes defender. The flowchart of the SEO algorithm is given in Figure 3.

## 4. Results and Discussion

The performance validation of the SEODTL-BDC model is carried out using benchmark breast ultrasound dataset [26]. It comprises 437 benign images, 210 malignant images, and 133 normal images. Some sample images are demonstrated in Figure 4.

Figure 5 illustrates a set of three confusion matrices produced by the SEODTL-BDC technique on the test dataset. The outcomes indicated that the SEODTL-BDC model has shown effectual classification under varying sizes of training/testing data. For sample, with training/testing data of 70 : 30, the SEODTL-BDC model has recognized 130 instances under benign class, 63 images under malignant class, and 39 images under normal class. Followed by, the SEODTL-BDC model has resulted in 174, 83, and 51 images into benign, malignant, and normal, respectively.

Table 1 provides the overall classification results of the SEODTL-BDC model on distinct training/testing data. The results outperformed that the SEODTL-BDC model has resulted in maximal classification performance under all training/testing dataset. For sample, with training/testing data of 50 : 50, the SEODTL-BDC model has offered average prec_*n*_ of 0.9903, reca_*l*_ of 0.9903, accu_*y*_ of 0.9949, and *F*_score_ of 0.9903. Simultaneously, with training/testing data of 70 : 30, the SEODTL-BDC model has provided average prec_*n*_ of 0.9891, reca_*l*_ of 0.9891, accu_*y*_ of 0.9943, and *F*_score_ of 0.9891. Concurrently, with training/testing data of 60 : 40, the SEODTL-BDC model has resulted in average prec_*n*_ of 0.9838, reca_*l*_ of 0.9815, accu_*y*_ of 0.9915, and *F*_score_ of 0.9827.

Table 2 and Figure 6 demonstrate a comprehensive comparative study of the SEODTL-BDC model with existing models on training/testing data of 50 : 50. The results indicated that the LD model has resulted in ineffectual outcome with the lower values of prec_*n*_, reca_*l*_, accu_*y*_, and *F*_score_. Besides, the ESKNN and FKNN models have reached slightly improved values of prec_*n*_, reca_*l*_, accu_*y*_, and *F*_score_. Along with that, the ESD and LSSVM models have obtained considerably increased values of prec_*n*_, reca_*l*_, accu_*y*_, and *F*_score_. However, the SEODTL-BDC model has accomplished superior performance with the prec_*n*_, reca_*l*_, accu_*y*_, and *F*_*score*_ of 0.9900, 0.9900, 0.9950, and 0.9900 correspondingly.

Table 3 and Figure 7 validate a wide-ranging comparative study of the SEODTL-BDC model with existing models on training/testing data of 70 : 30. The experimental values depicted that the LD model has led to worse performance with minimal values of prec_*n*_, reca_*l*_, accu_*y*_, and *F*_score_. In addition, the ESKNN and FKNN models have reached slightly improved values of prec_*n*_, reca_*l*_, accu_*y*_, and *F*_score_. Followed by, the ESD and LSSVM models have obtained considerably increased values of prec_*n*_, reca_*l*_, accu_*y*_, and *F*_score_. But the SEODTL-BDC model has outperformed the other methods with increased prec_*n*_, reca_*l*_, accu_*y*_, and *F*_score_ of 0.9840, 0.9820, 0.9920, and 0.9830 correspondingly.

Table 4 and Figure 8 exhibit a brief comparative study of the SEODTL-BDC model with existing models on training/testing data of 60 : 40. The experimental results portrayed that the LD model has reached ineffectual outcome with the lower values of prec_*n*_, reca_*l*_, accu_*y*_, and *F*_score_. Moreover, the ESKNN and FKNN models have reached certainly enhanced values of prec_*n*_, reca_*l*_, accu_*y*_, and *F*_score_.

Furthermore, the ESD and LSSVM models have obtained considerably increased values of prec_*n*_, reca_*l*_, accu_*y*_, and *F*_score_. However, the SEODTL-BDC model has reached better performance with the prec_*n*_, reca_*l*_, accu_*y*_, and *F*_score_ of 0.9840, 0.9820, 0.9920, and 0.9830 correspondingly.

Figure 9 inspects the comparative CT examination of the SEODTL-BDC with existing techniques. The results shown that the SEODTL-BDC technique has offered minimal CT over the other techniques under distinct sizes of training/testing data. For instance, on training/testing data of 50 : 50, the SEODTL-BDC technique has provided lower CT of 1.5130 m, whereas the ESD, LSVM, ESKNN, FKNN, and LD models have reached to higher CT of 3.3010 m, 2.0500 m, 3.1630 m, 2.1780 m, and 2.0150 m, respectively. Eventually, on training/testing data of 70 : 30, the SEODTL-BDC technique has offered reduced CT of 1.1420 m, whereas the ESD, LSVM, ESKNN, FKNN, and LD models have accomplished increased CT of 2.7850 m, 2.0100 m, 2.3620 m, 2.0720 m, and 2.1920 m, respectively.

Figure 10 demonstrates the ROC analysis of the SEODTL-BDC technique under different training and testing datasets. The figure exposed that the IAOA-DLFD system has reached enhanced outcome with the enhanced ROC of 98.4816 on training/testing (50 : 50).

The overall accuracy outcome analysis of the SEODTL-BDC method under training/testing (50 : 50) dataset is portrayed in Figure 11. The results demonstrated that the SEODTL-BDC technique has accomplished improved validation accuracy compared to training accuracy. It is also observable that the accuracy values get saturated with the count of epochs.

The overall loss outcome analysis of the SEODTL-BDC technique under training/testing (50 : 50) dataset is illustrated in Figure 12. The figure revealed that the SEODTL-BDC approach has denoted the reduced validation loss over the training loss. It is additionally noticed that the loss values get saturated with the count of epochs.

From the aforementioned tables and figures, it can be ensured that the SEODTL-BDC model has resulted in enhanced classification performance over the other methods.

## 5. Conclusion

In this study, a novel SEODTL-BDC approach has been developed for the detection and classification of breast cancer utilizing ultrasound images. The proposed SEODTL-BDC technique encompasses a series of subprocesses, namely, BF-based preprocessing, LEDNet-based segmentation, ResNet-18-based feature extraction, RNN-based classification, and SEO-based hyperparameter tuning. For demonstrating the improved outcomes of the SEODTL-BDC model, a sequence of simulations can be performed using benchmark dataset. Extensive comparative results pointed out the supremacy of the SEODTL-BDC approach over the existing methods. Therefore, the SEODTL-BDC model can be applied as a proficient tool for breast cancer classification utilizing ultrasound image. In future, advanced DL models can be utilized for enhanced breast cancer classification performance.

## Figures and Tables

**Figure 1:** Process of PAI.

**Figure 2:** Overall process of SEODTL-BDC technique.

**Figure 3:** Flowchart of SEO algorithm.

**Figure 4:** Sample images.

**Figure 5:** Confusion matrix of SEODTL-BDC technique under three training/testing datasets.

**Figure 6:** Comparative analysis of SEODTL-BDC technique under Training/Testing (50 : 50).

**Figure 7:** Comparative analysis of SEODTL-BDC technique under training/testing (70 : 30).

**Figure 8:** Comparative analysis of SEODTL-BDC technique under training/testing (60 : 40).

**Figure 9:** CT analysis of SEODTL-BDC technique under three training/testing datasets.

**Figure 10:** ROC of SEODTL-BDC technique under different training/testing datasets.

**Figure 11:** Accuracy of SEODTL-BDC technique under training/testing (50 : 50) dataset.

**Figure 12:** Loss of SEODTL-BDC technique under training/testing (50 : 50) dataset.

**Table 1:** Result analysis of SEODTL-BDC technique under distinct training/testing dataset.

Methods	Precision	Recall	Accuracy	*F*-score
Training/testing -50 : 50				
Benign	0.9954	0.9954	0.9949	0.9954
Malignant	0.9905	0.9905	0.9949	0.9905
Normal	0.9851	0.9851	0.9949	0.9851
Average	0.9903	0.9903	0.9949	0.9903
Training/testing -70 : 30				
Benign	0.9924	0.9924	0.9915	0.9924
Malignant	1.0000	1.0000	1.0000	1.0000
Normal	0.9750	0.9750	0.9915	0.9750
Average	0.9891	0.9891	0.9943	0.9891
Training/testing -60 : 40				
Benign	0.9943	0.9943	0.9936	0.9943
Malignant	0.9765	0.9881	0.9904	0.9822
Normal	0.9808	0.9623	0.9904	0.9714
Average	0.9838	0.9815	0.9915	0.9827

**Table 2:** Comparative analysis of SEODTL-BDC technique with recent approaches under training/testing -50 : 50.

Methods	Precision	Recall	Accuracy	*F*-score	Classification time (m)
SEODTL-BDC	0.9900	0.9900	0.9950	0.9900	1.5130
ESD model	0.9880	0.9880	0.9890	0.9880	3.3010
LSVM model	0.9890	0.9890	0.9890	0.9890	2.0500
ESKNN model	0.9860	0.9660	0.9870	0.9860	3.1630
FKNN algorithm	0.9870	0.9870	0.9870	0.9870	2.1780
LD algorithm	0.9860	0.9860	0.9860	0.9860	2.0150

**Table 3:** Comparative analysis of SEODTL-BDC technique with recent approaches under Training/Testing -70 : 30.

Methods	Precision	Recall	Accuracy	*F*-score	Classification time (m)
SEODTL-BDC	0.9890	0.9890	0.9940	0.9890	1.1420
ESD model	0.9820	0.9830	0.9900	0.9820	2.7850
LSVM model	0.9810	0.9790	0.9910	0.9810	2.0100
ESKNN model	0.9800	0.9810	0.9810	0.9800	2.3620
FKNN algorithm	0.9770	0.9770	0.9770	0.9770	2.0720
LD algorithm	0.9760	0.9760	0.9770	0.9760	2.1920

**Table 4:** Comparative analysis of SEODTL-BDC technique with recent approaches under training/testing -60 : 40.

Methods	Precision	Recall	Accuracy	*F*-score	Classification time (m)
SEODTL-BDC	0.9840	0.9820	0.9920	0.9830	1.0920
ESD model	0.9870	0.9860	0.9870	0.9870	1.5720
LSVM model	0.9850	0.9850	0.9860	0.9850	1.1470
ESKNN model	0.9800	0.9790	0.9800	0.9800	1.3220
FKNN algorithm	0.9780	0.9780	0.9780	0.9820	1.4090
LD algorithm	0.9810	0.9810	0.9810	0.9840	1.4220

## Data Availability

Data sharing not applicable to this article as no datasets were generated during the current study.
